# Biosynthesis of Iron Oxide Nanoparticles Using Leaf Extract of Ruellia tuberosa: Mechanical and Dynamic Mechanical Behaviour Kevlar-Based Hybrid Epoxy Composites

This article has been retracted.

**DOI:** 10.1155/2023/1731931

**Published:** 2023-04-20

**Authors:** L. Natrayan, Yenda Srinivasa Rao, Gayatri Vaidya, Sumanta Bhattacharya, S. Kaliappan, Pravin P. Patil, Prabhu Paramasivam

**Affiliations:** ^1^Department of Mechanical Engineering, Saveetha School of Engineering, SIMATS, Chennai 602105, Tamil Nadu, India; ^2^Department of Mechanical Engineering, Sri Sivani College of Engineering, Srikakulam, Andhra Pradesh, India; ^3^Department of Studies in Food Technology, Davangere University, Davangere, Karnataka, India; ^4^Department of Textile Technology, Maulana Abul Kalam Azad University of Technology (MAKAUT), Westbengal, Kolkata, India; ^5^Department of Mechanical Engineering, Velammal Institute of Technology, Chennai, Tamil Nadu, India; ^6^Department of Mechanical Engineering, Graphic Era Deemed to be University, Bell Road, Clement Town 248002, Dehradun, Uttarakhand, India; ^7^Department of Mechanical Engineering, College of Engineering and Technology, Mettu University, Metu 318, Ethiopia

## Abstract

One of the more enticing, ecologically responsible, as well as safe and sustainable methodologies is eco-friendly nanomaterial synthesis. Vegetation materials will be used as reductants instead of toxic substances for synthesising nanoparticles. The current study used Ruellia tuberosa (RT) leaf extract digest to synthesise FeO nanomaterials, which were then characterised using XRD. Following that, microbially produced FeO molecules were mixed with a Kevlar-based polymeric matrix to study the blended consequences. To examine the interbreeding, the current experimental analyses were performed, including both static and dynamic mechanical characteristics. The addition of FeO nanofillers improved the elastic modulus, tensile strength, and storage modulus of the nanocomposite. Impact force uptake has been raised to a certain extent by the addition of nanoparticles. The findings of this research show that incorporating FeO nanofillers into Kevlar fabrics is a promising technique for increasing the mechanical characteristics of hybrid laminated composites. As per DMA evaluation, the sample without nanomaterials had a more volcanic lava response, which is a useful thing for body systems for missile use. Another critical aspect of a nanoparticles-filled nanocomposite that must be addressed is the relatively uniform scattering of padding as well as the development of interfacial adhesion in such a combination. The presence of FeO fillers in polymeric composites is confirmed by XRD analysis.

## 1. Introduction

Nanomaterials seem to be a promising as well as rapidly expanding scientific discipline that is trying to fill shortfalls in contemporary advanced components. Nanoscience has also advanced in the sector of nanotechnologies over the last two decades. Nanomaterials (NPs) are fine pieces with diameters varying from 0 to 100 nm [1]. The compositional distinctiveness of NPs, such as diameter, structure, and fractal, has also enhanced their use in digital equipment, biomedicine, pharma, and textile manufacturing, as well as biological markers and biosensing. The intersection of chemical synthesis as well as nanotechnology opens up an amazing new frontier for the creation of sustainable and clean multipurpose nanomaterials [2, 3]. Aside from precious metals, bioactive synthesis of metal nanoparticles has already been expanded to a variety of metal oxides with intriguing properties. Multipurpose nanocrystals (IONPs) have also emerged as a potential substance with implementations in bioengineering, skincare, phytoremediation, and diagnostic tools, as well as fabrication techniques. Moreover, the use of IONPs in biology and medicine is expanding rapidly. IONPs have heretofore proven to be extremely capable of sustained release for muscle repair as well as therapeutic interventions for tumours. Because of its perfect materials with high surface, tiny group disparity, as well as consistency, it has a wide spectrum of uses [4, 5].

Among various NPs, metal oxide NPs have been regarded as safe for people and wildlife. The essential metallic category has applications in electrochemical processes and conservation biology, as well as magnetisation physiology. Between nanostructured materials, iron oxide (FeO) is by far the worthiest of mention because it is resorbable and has magnetism that aids in treating diseases and diseases [6, 7]. Iron oxide nanoparticles (IONPS) have a wide range of applications, including catalysts, hard rock adsorbents, colourants, and antibacterial drug deterioration. Participants have antibacterial activities against pathogenic microbes. The traditional treatments that use it for nanoparticle synthesis are the significant problems with IONPs [8]. Physicochemical formulation encompasses the use of costly and hazardous substances as limiting as well as reductants. The use of dangerous and toxic chemicals will have a negative impact on healthcare as well as biomedical applications.

Given the drawbacks of traditional chemical methods, quasibiomaterial, as well as ecologically responsible strategies for nanoparticle synthesis can be achieved by the use of biomass entities. Seedlings, phytoplankton, microorganisms, and pathogens have previously been used as biomass entities, but use of seedlings is now widespread [9, 10]. Crops have an abundant supply of phytonutrients like amino acid residues, carbs, flavones, nutrients, tannins, terpenes, and nucleophiles, as well as total sugars. In metal sodium chloride, metal ions are reduced to metallic ions during the biosynthesis pathway of NPs. The above-given preliminary decrease creates a precipitate centre point, which leads to a sequester of extra metallic ions as well as integrates the adjoining precipitate location [11]. The creation of nanomaterials is caused by the end state. The NPs are integrated into vegetation biomolecules, which also retain consistency as well as enhance morphological characteristics. The nontoxic nature of biosynthesized NPs has displaced traditional chemical NP synthetic routes. The metal NP biosynthesis pathway is a cheap, nontoxic, and straightforward method of NP synthesis. The oxidising agents used for the nps synthesis are nontoxic and ecologically responsible [12]. The number of scientific academic publications utilising seedlings as well as their different bits demonstrates in the above-given theory.

Nanomaterials are created using a variety of chemical methods. Thermal degradation, geothermal formulation, microemulsions, founder, segments and subtechniques, sol-gel synthesising, father chemical, and pyrolysis as well as hydroxylation of catalysts, ionisation synthesising, and high performance liquid synthesis, as well as flocculation science techniques are all used in the synthesis of IONPs [13, 14]. The scattering as well as homogeneity of magnitude and crystalline size have been poor for certain methodologies like the solvothermal method as well as the sol-gel procedure. Despite these disadvantages, IONPs were synthesised using liquid-like metal salts, hydrazine, and sodium dodecyl sulphate. Toxic sludge flows from those kinds of biological fabrication techniques can be harmful to society. Such synthetic paths increase the likelihood of nanomaterial aggregation [15, 16]. Similarly, physiological synthesis implies are frequently expensive due to their energy requirements. Until now, such physical processes have been efficient in synthesis; however, there should be a fundamental shift forward in low-cost, stable, colored, and environmentally friendly IONP synthesis methodologies [17, 18]. Different biochemical assets, such as phytoplankton, microorganisms, microbes, and crops, have also surfaced as premium and environmentally friendly portals for synthesising nanoparticles. Many investigators have been drawn to the interaction of traditional medicines and bioactive nanostructures in order to create nanocrystals for a variety of applications. Due to their rich phytochemical as well as phytochemical constituents, medicative species are commonly used and favoured again for the production of nanomaterials [19, 20].

Numerous vegetation extracts have been evaluated so far for the synthesis of IONPs. Overall, metallic nanoparticles have antibacterial properties and the ability to degrade contamination. It can also be used to avoid microbial pollutants in fabrics, polymers, as well as other diagnostic implants. In contrast to many other nanostructured materials, IONPs have those kinds of benefits [21, 22]. The use of IONPs is a substitute for using fungicidal agents to handle pathogens. Aside from that, IONPs can indeed be efficiently removed or excluded by using magnetism. The current research was the first one to disclose mostly the synthesis of IONPs utilising R. tuberosa leaf extract [23]. A. tuberosa, also known as Mimi rhizome or Chipset rhizomes, is a member of the Acantharean community, which is plentiful in Asian countries. R. tuberosa leaf was shown to have antitumor activity, antibacterial, as well as anti-inflammatory characteristics [24].

Numerous scientists have created nanocomposite by incorporating natural materials like wood fibres as well as natural materials such as fibres into adhesives, synthetic fibers, polyphenol, polyvinylidene ester, and methacrylate isocyanate polymers. As a substitute for synthetic fibres, environmentalism drew researchers to create fresh nanocomposites with the addition of much more than a reassurance from natural assets, such as plant fibres or synthetics made from natural amendments [25, 26]. The mixture of nanofiller as well as organic fibre in the composite leads to decreased moisture absorption as well as enhanced structural characteristics. These kinds of facts are depicted in different research. The increase in the content of bentonite improves the mechanical characteristics of husk semolina-polypropylene blends [27]. While contrasted to certain other naturally derived fibres, Kevlar has several desired traits that also provide it a strong position in a variety of massive numbers of applications. Its most essential feature has been its good strength. That also implies it will have excellent mechanical properties at a lower weight than traditional materials [28].

Although Kevlar is steady for most chemical forms, this can degrade once revealed to certain soluble enzymes, foundations, or hypochlorite. Investigations have indicated that it should be used as a metal replacement because it is nearly significantly more powerful. Once crocheted as well as knitted with a 50% structure of Kevlar as well as polypropylene fabrics, the compounds demonstrated significantly greater cut tension indicator, suitable for use in activewear as well as medical uses [28, 29]. Numerous studies and research have been conducted on the advancement of Kevlar in protective gear uses as well as the optimization of the requisite material properties. A few studies have concentrated on maximising the components in blends in order to obtain the desired qualities while minimising poundage. As a hopeful field of research, there is much to be done in terms of production, experimenting, as well as the atmosphere wherein the merchandise is used. As a result, this report provides a summary of certain research articles on Kevlar-based synthetic structures [30].

The main objective of this research is to assess the mechanical performance of bio-synthesised IONPs made from R. tuberosa leaf extract mixed with Kevlar fibre. The nanocomposite was created using compression moulding techniques to achieve the aforementioned goals. Following fabrication, the composites were tested and the influence of the prepared nanoparticle filler was evaluated using the standard specifications. The XRD patterns have been used to indicate the existence of IONPs particulate.

## 2. Materials and Methods

### 2.1. Materials

Sekar Fibrous Materials Ltd., Coimbatore, Tamil Nadu, India, supplied the Type 29 Kevlar fibre mat. Abi Tech Chemicals in Coimbatore supplied the ferrous sulphate and sodium hydroxide. Plant samples were obtained from the National College of Engineering in Kovilpatti, Tamil Nadu, India.

### 2.2. Bio Synthesis of FeO Nano Materials

The vegetation samples were cleansed with deionized water to remove contaminants and dust that had accumulated on the plant parts. The tuberosa sapling's leaves have been trimmed as well as detached. 10 g of leaves have been cut as well as cooked in 120 ml of distilled water for 15 minutes at 60°C. The resulting mixture has been collected and kept at 5°C for even further assessment after the solvent has been sifted. For this response, ferric sulphuric acid (1M) was employed as a forerunner. Ferric sulphate has been mixed with Ml of pure water to make it. A total of 300 mL of pure water has been added to 55 mL of leaf supernatant. The plant material (55 mL) and Na_2_CO_3_ pellets (2 g) were added to a 55 mL ferric chloride solvent. After centrifuging the combination, the supernatant was removed. The brownish black canister has been left to dry as well as store it for further research.  Figure 1 shows the bio synthesis process of FeO formations [10].

### 2.3. Preparation of FeO/Kevlar Based Nano Composites

Compression moulds with scientific equipment were used to create polymeric specimens. The moulded heat was 250°C. The deformation was just very low (approximately 1.30 bar), but the mould duration was really quite long (30 min). The production settings were chosen to achieve maximum pellet aggregation while minimising material movement. The bio-synthesised FeO particles in various concentrations had been deeply sonicated with epoxy matrix prior to compression moulding. The mixture was then poured into a Kevlar fibre mat with dimensions of 150 × 150 × 3 mm. Finally, the prepared mould was placed in the compression moulding machine at the temperatures and pressures specified. In reality, while the manufacturing process usually results in ideal aggregation, thermoplastic flow may be to blame again for performance degradation for nanomaterials. In the moulding process, mould temperature and duration could be enhanced to decrease movement of materials without impacting pellet aggregation. To prevent an oxidation reaction, mould pressure must be lowered.

### 2.4. Characterization of FeO-Based Nano Composites

Tensile properties were conducted at ambient conditions and 50% humidity levels. The tensile test was executed in accordance with the ASTM requirement D 638-03. A UTM with a 50 kN strain gauge was employed in this research. Tension tests were carried out with a crosshead dragging at a rate of one millimetre per minute till the samples failed. Flexing experiments were also performed at ambient conditions and 50% humidity levels. For every polymeric type, specimens to measurements of 125 × 12 × 3 mm were evaluated in accordance with the ASTM D790 requirement. The Charpy impact test method was employed to determine the impact durability of the composite specimens in accordance with ISO 179. The Dynamic Mechanical Analyzer was used to examine the dynamic mechanical characteristics. The X-ray scattering graphs have been captured to use an X-ray spectrometer at 30 kV as well as 25 mA execution capabilities. The X-ray diffraction pattern was screened to 2.5 A radioactivity as in 2 range of 10−80° to 0.02 stages at a monitoring rate of approximately two degrees per minute.

## 3. Result and Discussions

### 3.1. X-Ray Diffraction

An X-ray interference pattern (XRD) uses X-rays to determine the geometric features or frame of a particle. The elastically scattered X-rays from the atomic nuclei do have a lengthy sequence.  Figure 2 shows the X-ray scattering spectroscopy of the biologically synthesised FeO annealing temperature at 500°C in an outdoor area heater. The identified Bragg peaks matched the pure (Fe_2_O_3_) tetrahedra textures. The lattice parameters were calculated to be equal to 8.24000 A° and equal to 24.02000 A°. (210, 204, 206, 207, 215, 106, and 115) crystalline representations imply a crystalline phase of FeO particles. The two theta stances are 31, 32.5, 28.96, 29.15, 21.50, and 34.56. It should be noted that montmorillonite as well as hematite seem to be tetrahedral, which implies that the XRD method could indeed distinguish among them, particularly in the nanostructured region, in which the character trait representations seem to be broad as well as seem to occur almost simultaneously in the two places. The highs' locations have been compared on a 2 level with previous reports, and their locations have been discovered to be very similar. There were no further elements discovered until the point of the XRD pattern, demonstrating the purity of biomimetic FeO nanostructures [31–33].

### 3.2. Mechanical Properties

#### 3.2.1. Tension Behaviour

The ductility of blended fabricated composites made from various fractions of FeO nanomaterial was also studied, and the results are depicted in Figure 3. Originally, the inclusion of FeO nanomaterials enhanced the tensile characteristics of the specimen by up to 5%. As shown by combination nanocomposites with 7.5% FeO nanomaterials, enhancing the amount further than this point reduces the ductile quality of the specimen. It is possible to conclude that at 5% accumulation, there is really unified scattering and dispersion of nanofillers inside the mixture as well as materials [34]. It results in a kind of a unified packing dispersion between the matrix and the filler, which improves the laminate's elastic modulus. There is a strong temptation for nanomaterial aggregation with such a higher proportion of nanofillers (7.5%). The reduction in interfacial bonding was ultimately caused by such aggregates. It eventually caused the material's strength to deteriorate. Increased nanomaterial concentration has also occurred, contributing to the weakening of nanocomposites [35]. The inclusion of FeO nanomaterial increased the composite's elastic strength, as seen in Figure 3. When compared to plain epoxy, the 5 wt.% and 7.5 wt.% FeO-filled composites improve strength by 73.12% and modulus by 55.93%.

The yield strength, or modulus, is a characteristic of matter that is determined by the comparative portion of components. The biocomposite materials contain a presence of fillers. As the FeO nanoparticles stiffen, the yield strength increases. This rise is consistent with an increment in nanofillers. Using the principle of blends, a similar phenomenon could be anticipated. The toughness characteristics observed from the stress-strain graph for additional support the rise as well as the consequent reduction in strength properties. Following that, extra tiny peaks appear inside the matrix as strain increases, with such a pointed variance at ultimate load, most probably portraying the inability of certain fibres. The polymeric sample type A as a whole appears to have yield strength [36]. According to our previous theory, introducing 5% FeO nanoparticles enhanced composite toughness, which is affirmed by the typical stress-strain curve. When contrasted to composite A, the preliminary deformation owing to crack formation was measured at 249 MPa. The above-given pattern's rupture behaviour is also durable, with a number of minor highs prior to actually defeat. However, in the particular instance of D type, the peak diversion is nearly the highest.

#### 3.2.2. Bending Behaviour

Once confined to a bending load, the flexural test regulates the most intensive process inside the composites prior to actually fracturing or breaking. The experiment consists of a rectangle bar supported by two aids and packed through a trying to load nose located currently halfway between endorses. The area beneath the flexing nasal passages is very small, and strain is concentrated only at the head, resulting in breaking here.  Figure 4 depicts the flexural variability for laminated structures containing 0, 2.5, 5, and 7.5% FeO nano fillers. The findings reveal that the addition of nanofillers enhanced the flexural resilience of the composite specimens substantially. The flexural strength increased as that of the padding weight percentage increased. The addition of fillers increased interfacial interactions, which led to an increase in flexural strength. The flexural techniques to be evaluated also demonstrate an increase in interfacial interaction. The governed specimen has much more deformation, which is reduced by adding FeO fillers [37]. There seems to be no substantial improvement in flexural strength when the packing is increased by more than 5%. It implies that its particulate loading impact contributes to flexural as well. It is being discovered to increase rubbing between flanges as well as reduce flexural strength. The presence of filler particles also had an impact on the flexural modulus of blended lightweight materials. As a consequence, rigidity and flexural toughness have been enhanced, despite the lack of a significant difference in flexing elastic properties at 5 and 7.5% loading rates. This one is explained in the context of padding scattering as well as interfacial bonding in the mixture [38]. The bending and tensile performance indicate that interfacial bonding has a significant effect on resilience, whereas yield strength is much more impacted by the rigidity of its components. When compared to plain epoxy, the 5 wt.% and 7.5 wt.% FeO-filled composites improve flexural strength by 51.69% and modulus by 67.31%.

#### 3.2.3. Charpy Impact Properties

Impact examination, professionals use impact testing to anticipate how a substance will behave under realistic conditions. Numerous components fail unexpectedly when struck, usually at faults, fissures, or gouges.  Figure 5 depicts the findings of a Charpy test assessing the in-plane fracture toughness of biocomposites. The impact velocity was measured at 2.5 m/s at a uniform speed, and the percussion material and decline angular position used were 5.26 kg and 121.58, respectively [39]. An increase in nanoparticle concentration of up to 5% resulted in an increment in impact resistance, implying that the nanofiller packed nanocomposite has a highly energetic absorption capacity. The impact strength decreased with a high amount of FeO nanofiller. Such an action is related to that of the composite material in tension tests, presumably due to filler particle aggregation containing high concentrations. When compared to plain epoxy, the 5 wt.% FeO-filled composites improve impact strength by 57.36%.

### 3.3. Dynamic Mechanical Analysis

Throughout this research, dynamic mechanical analysis (DMA) of composite materials at various padding loadings was conducted to examine the variability of storage modulus (E1), loss modulus (E11), as well as dissipative component (Tan X). Formula (1) illustrates its correlation:

(1) $$\begin{array}{c} Tandelta=\frac{E11}{E1}\text{.} \end{array}$$

Figures 6(a)–6(c) show the storage modulus, loss modulus, and tan delta, as well as tan delta maximum virtues of prepared specimens obtained by plotting against heat. The temperatures ranged from ambient temperature to 160 degrees Celsius, and indeed, the changes in such variables were registered.  Figure 6(a) shows how the storage modulus virtues altered even as the particulate packing ratio was increased. Storage modulus has been higher with higher nanoparticle concentration than at lower filler packing. This was due to filler's improved ability to engross energy [9]. As a result, the particulate mass flow straightened the composite's load bearing capacity. In contrast to blended nanocomposites with nanoparticles, the composite made without nanoparticles had the minimum storage modulus valuation. This behaviour is similar to that of nanocomposite in fixed tension tests, in which a demonstrated the smallest elastic moduli values as well as D demonstrated the greatest [26]. Moreover, as seen in Figure 6(b), the loss factor increased with increasing particulate volume fraction. A nanocomposite with a higher electron loading of 7.5% seemed to have the greatest loss modulus, which reduced as the proportion of particulate introduced inside the specimen reduced. Tan delta is obtained by plotting against heat in Figure 6(c). This is a virulent acceleration response proportion. The Tan delta has the tallest mountain at a particulate loading of nil, implying that it is more hygroscopic than nanomaterials [40]. The substance was becoming stretcher in specimens of nanomaterials with nanoparticles even as the proportion of a filer was enhanced, and when a load is applied, it has a greater capacity to store the pile. The tan delta rises in value as the nanomaterial loading increases. This suggests that the substance has a more viscous reaction even though nanostructures start creating constraints inside of substances again for movement of polymerization, resulting in a more viscoelastic reaction.

## 4. Conclusion

The inclusion of bio-based FeO nanofiller provides several benefits, including a tensile strength of approximately 5% particulate prefetching. This same inclusion of more nanoparticles lowered the mechanical properties but enhanced the elastic modulus all across the whole loading rate additament.

- The modulus of elasticity as well as elastic moduli outcomes showed comparable behaviour. The inclusion of bio-based FeO nanomaterials increased the inherent quality of the composites by up to 5%. The inclusion of more nanoparticles reduced the impact force uptake. Moreover, because of the inclusion of rigid fillers, the inclusion of nanoparticles altered this same content's failure behaviour from brittle fracture.
- When compared to plain epoxy, the 5 wt.% and 7.5 wt.% FeO-filled composites improve strength by 73.12% and modulus by 55.93%. At the same time, it shows an improvement in flexural strength by 51.69%, modulus by 67.31%, and impact strength by 57.36%.
- According to DMA experiment, the specimen without nanoparticles exhibited a more pyroclastic reaction, which is a desired feature for structures of the body for projectile usage. Whereas impact resistance as well as tensile modulus were increased to some level with nanoparticle loading, this same impact on engineering properties is showing promise. As a consequence, fresh research is required, including identifying the crucial peak where the tensile strength as well as impact assimilation begin to decline.
- Another crucial element of nanofiller packed nanocomposite that must be discussed is the relatively homogenous scattering of padding as well as the development of its crosslink density with such a mixture. The existence of FeO filler particles in the polymer matrices is confirmed by XRD analysis.

## Figures and Tables

**Figure 1:** Bio-synthesis of FeO from Ruellia tuberosa leaves.

**Figure 2:** XRD pattern of FeO/Kevlar/epoxy based hybrid composites.

**Figure 3:** Tensile strength and its modulus of FeO/Kevlar/epoxy based hybrid composites.

**Figure 4:** Bending strength and its modulus of FeO/Kevlar/epoxy based hybrid composites.

**Figure 5:** Impact strength of FeO/Kevlar/epoxy based hybrid composites.

**Figure 6:** Temperature vs storage modulus, loss modulus and tan delta.

## Data Availability

The data used to support the findings of this study are included within the article. Should further data or information be required, these are available from the corresponding author upon request.
